RETRACTED

# A Novel Necroptosis-Related lncRNA Signature for Osteosarcoma

**DOI:** 10.1155/2022/8003525

**Published:** 2022-07-07

**Authors:** Yixin Zheng, Jie Xu, Jiexiang Lin, Yuan Lin

**Affiliations:** ^1^Department of Orthopaedics, Fujian Provincial Hospital, Fuzhou 350001, China; ^2^Shengli Clinical Medical College of Fujian Medical University, Fuzhou 350001, China

## Abstract

**Backgrounds:**

Osteosarcoma (OS) is easy to metastasis. Necroptosis-related long noncoding RNA (lncRNA) (NRlncRNA) plays a vital role in the tumorigenesis of many malignant tumors. Nonetheless, there have been few studies investigating the relations between NRlncRNA and OS. During the investigation, NRlncRNAs in OS were confirmed and characterized and their relationships with prognoses were investigated.

**Methods:**

NRlncRNAs were downloaded from The Cancer Genome Atlas (TCGA) OS expression data and clinical-pathological information. First, univariate Cox regression and LASSO regression analyses were used to screen for prognostic-related NRlncRNAs. Second, multivariate regression analyses were used to establish a prognostic nomogram for predicting individual survival probability. Survival analyses demonstrated that high-risk patients (HRPs) had a poor prognosis. In addition, gene set enrichment analyses (GSEA) were used to identify gene function in high- and low-risk groups based on the survival mode.

**Results:**

The 7 NRlncRNAs (AC004812.2, AC022915.1, AC073073.2, AC090559.1, AL512330.1, DDN-AS1, and SENCR) were shown to have a distinct difference and were used to construct an NRlncRNA signature. Using the signature as a risk score was an independent factor for OS patients. The signature divided OS patients into the high- and low-risk groups. Furthermore, the seven lncRNAs were significantly enriched in cell migration and metabolism.

**Conclusions:**

The 7 NRlncRNA survival models have the potential to serve as therapeutic targets and molecular biomarkers for patients with OS, as well as to precisely predict OS prognoses.

## 1. Introduction

Osteosarcoma (OS) is a common primary malignancy of the bones. The remaining therapeutic challenge and poor prognosis for OS is metastasis [1]. Smeland et al. reported that metastasis and tumor position are two significant factors highly associated with poor prognoses of OS patients [2], while incomplete surgical resection and poor response to chemotherapy also result in poor prognosis [3]. Increasing the survival rate of OS patients has been shown to be difficult for a long time, although the treatment for this disease is on the verge of being developed [4].

Necroptosis can be thought of as an alternate model of programmed cell death, and it also plays a role in oncogenesis and cancer metastasis [5]. In the past few decades, numerous studies on OS necroptosis have been conducted [6–8]. Consequently, finding a gene set related to necroptosis is essential for predicting OS prognoses.

RETRACTED

Although long noncoding RNA (lncRNA) cannot encode proteins [9], it is the key to cancer occurrence and development [10–13]. Currently, studies show that necroptosis-related lncRNAs (NRlncRNAs) are associated with poor prognoses in a variety of tumors, including lung adenocarcinoma, gastric cancer, breast cancer, and head and neck squamous cells. However, the function of NRlncRNAs in OS and their association with patient prognosis remain unknown [14–17].

It is imperative to screen necroptosis lncRNA associated with OS prognoses. In this study, NRlncRNA was screened for and examined in a lncRNAs' expression dataset in OS from TCGA. The NRlncRNA signature was validated for predicting OS patient survival outcomes.

## 2. Materials and Methods

### 2.1. OS Patient Data

The RNA sequencing (RNA-seq) data and clinical data of OS patients were obtained from TCGA database (https://cancergenome.nih.gov/). In this study, data from 383 OS patients were analyzed. The exclusion criteria for the samples were (1) the loss of clinical and follow-up information and (2) the presence of other malignancies. Finally, 85 patients were included in this study.

### 2.2. Screening of Necroptosis-Associated Genes in OS

Genes associated with necroptosis were screened from the Kyoto Encyclopedia of Genes and Genomes (KEGG) (https://www.kegg.jp), and a total of 159 necroptosis-related genes were obtained. The GENCODE annotation file was used to identify 3223 lncRNAs in TCGA in combination with the GTEx datasets (http://cance rgeno http://me.nih.gov/about tcga). Pearson correlation algorithm was used to identify necroptosis-associated DE lncRNA with ∣*R*^2^ | >0.3 and *P* < 0.001. After completing the screening process, 65 NRlncRNAs were obtained for further analyses using the limma package in R.

### 2.3. Analysis of NRlncRNA Prognostic Signatures for OS

Univariate Cox proportional hazard analyses and Kaplan-Meier analyses were used to determine the association between NRlncRNA and OS survival, and *P* < 0.01 was incorporated into the least extreme shrinkage and selection operator (Lasso) regression. Multivariate Cox proportional hazard analyses were performed to establish the best prognostic risk model using the R survival package, and the risk score (RS) was determined using the formula: risk score = *Σ*_*ⅈ*=1_^*n*^*β*_*i*_∗(expression of lncRNA_*i*_) [13]. The OS patients were classified into two groups based on the median RS: low- and high-risk groups. Kaplan-Meier survival analyses were used to estimate the survival differences between the two groups in the R survival package.

RETRACTED

### 2.4. Modeling of Prognosis

Multivariate and univariate Cox analyses were performed to determine the association between survival prognoses with clinical considerations (CFs) and RS using the R survival package. The survival ROC R package was used to generate time-dependent receiver operating characteristic (ROC) plots for measuring the predicted accuracy for survival time across various CFs and RS. The R rms package was used to construct a nomogram containing RS and CFs such as age, stage, and gender. The nomogram predicted the one-, three-, and five-year survival of OS patients. The R survival package was used to plot the nomogram calibration curve. The calibration curve demonstrated the nomogram's predictive ability.

### 2.5. Statistical Analysis

The survival plots were generated using Kaplan-Meier methods, while the log-rank test was used for comparison. The Lasso and Cox regression methods were used to estimate the prognostic effect of clinicopathological data and the NRlncRNA signature. Statistical analysis was carried out using the R language. An analysis of bilateral data was conducted, and *P* ≤ 0.05 was considered statistically significant. Gene set enrichment analysis was used to perform the functional annotation (GSEA, http://www.broadinstitute.org/gsea/index.jsp), and the top five KEGG pathways and Gene Ontology (GO) terms associated with necroptosis have been identified, as well as the functional enrichment of NRlncRNAs with prognostic value.

## 3. Results

### 3.1. NRlncRNA with Prognostic Value in OS

When necroptosis-associated RNA and lncRNA coexpression networks were combined, 3223 NRlncRNAs were obtained. Kaplan-Meier analyses and Cox proportional hazard analysis demonstrated that 58 NRlncRNAs from TCGA were significantly associated with OS patient survival (*P* < 0.01). Using Lasso analysis, 13 NRlncRNAs were discovered to be precisely associated with OS patient survival. Furthermore (Figure 1), multivariate Cox analyses identified 7 lncRNAs with prognostic significance, including 1DDN-AS1, AC022915.1, AC090559.1, AL512330.01, SENCR, AC073073.2, and AC004812.2 from the 13 NRlncRNAs (Table 1). A visual coexpression network of NRlncRNA-mRNA was constructed using the 7 lncRNAs as the best prognostic risk model (Figure 2) was established.

Calculated according to the risk score formula, the median risk score was used to categorize the patients into two groups: high-risk and low-risk groups. The log-rank test was used to compare the overall survival rates between the two groups. The overall survival of the high-risk group was lower than the low-risk group (Figure 3(a)). Furthermore, four lncRNAs (AC022915.1, AC090559.1, AC073073.2, and AC004812.2) were favorable prognostic factors, and the others (DDN-AS1, AL512330.1, and SENCR) were harmful prognostic factors (Figures 3(b)–3(h)).

RETRACTED

### 3.2. Evaluation of the OS Patients' Survival

Univariate and multivariate Cox regression analyses were performed to determine the independent prognostic factors (IPFs) of OS. By univariate Cox regression analysis (UCRA), the RS had a hazard ratio (HR) of 1.038 (95% CI 1.023−1.053) (*P* < 0.001). By multivariate Cox regression analyses (MCRA), risk score remained independent even after controlling clinical features (HR = 1.050, 95% CI 1.031−1.070) (*P* < 0.001) (Figures 4(a) and 4(b)). The area under the ROC curve for RS (AUC) was 0.961, compared to those of other clinical factors (Figure 4(c)), indicating that the 7 NRlncRNAs were suitable for the OS prognostic risk model. The risk score, metastasis, and gender were used to establish a nomogram to predict survival in OS patients (Figure 5). Based on the ROC plot, the areas under the one-, three-, and five-year survival lines were, respectively, 0.903, 0.907, and 0.903(Figure 6(a)). The calibration plot exhibited excellent nomogram prediction ability, and the C-index of the prognostic model was 0.797 (0.761-0.833) (Figure 6(b)).

### 3.3. GSEA Enrichment

GO analyses revealed that NRlncRNA was significantly enriched in cell-matrix adhesion. The KEGG pathway analyses revealed that NRlncRNA was significantly enriched in focal adhesion, regulation of action cytoskeleton, and metabolic processes (Figure 7).

## 4. Discussion

Osteosarcoma is an aggressive and life-threatening bone tumor. In patients with OS without metastasis, the five-year survival rate is approximately 70%. However, when accompanied by distal metastases, it decreases to 20% [18]. Therefore, it is important to identify biomarkers that can predict the prognoses of OS patients. There are some NRlncRNAs that can be used as prognostic biomarkers for cancer. They are capable of regulating tumor progression and metastasis [19]. Consequently, it is necessary to establish an NRlncRNA signature to predict OS prognoses. It is our knowledge that this is the first study to establish a risk model based on NRlncRNA for predicting patient outcomes in OS.

In this study, 58 prognostic NRlncRNAs were confirmed through analyses of public RNA sequence data. Multivariate Cox proportional hazard analysis and LASSO Cox regression analyses revealed that 7 NRlncRNAs (AC004812.2, AC022915.1, AC073073.2, AC090559.1, AL512330.1, DDN-AS1, and SENCR) were strong candidates for use as prognostic markers. For one, three, and five years of survival, the areas under the ROC curve were 0.903, 0.907, and 0.903, respectively. The outcome suggested that the risk score signature could predict survival. Based on the ROC plot outcomes, the AUC of the RS established using the 7 NRlncRNAs was 0.961, which was superior to the current index (such as gender, metastasis, and metastasis site) for predicting prognosis. In the NRlncRNA model, we discovered that HRPs had much worse outcomes than low-risk patients. Based on the results of the calibration curve, ROC curve, and C-index, the model exhibited greater accuracy and discrimination, indicating it could serve as a feasible approach for predicting OS in patients.

RETRACTED

GSEA revealed a close association between NRlncRNA and cell-matrix adhesion. Cell-matrix adhesion plays a major role in biological processes, such as gene expression regulation, survival, differentiation, proliferation, and cell motility. Focal adhesions were formed in the cell-extracellular matrix microenvironment. Some fragment of focal adhesions contributes to the formation of the link between the actin cytoskeleton and film receptors. Multimolecular complexes that connect plaque proteins anchor actin filaments to transmembrane receptors of the integrin family. Other fragments of focal adhesion consist of signal molecules such as protein kinase, phosphatase, their substrates, and other adapter proteins. The integrin signaling pathway is highly dependent on the nonreceptor tyrosine kinase activities and adaptor protein functions to initiate downstream signaling events, such as FAK, src, and Shc proteins. Finally, the actin cytoskeleton is reorganized as a result of these signaling events.

Numerous studies demonstrated that adhesion, which is mediated by focal adhesion points on the substrate, has long been regarded as a crucial step in cell migration. Inadequate migration can result in cancer metastasis [20], while the precise coordination of actin cytoskeleton movement is required for tumor metastasis [21]. To achieve metastatic regeneration, the remodeling of the extracellular matrix (ECM), the activation of downstream signaling pathways, and the precise coordination of actin cytoskeleton dynamics are essential to enable cancer cells to respond to external cues and to define the complex invasion and metastasis potential of cancer cells [21, 22].

Nonetheless, there are several limitations of our research. Firstly, the sample size might be not large enough for generalizing the conclusions. Secondly, the data used for analysis is only collected in TCGA, in order to better understand the value of the signature in vivo, clinical trials are required.

RETRACTED

## 5. Conclusion

To conclude, we developed and validated a novel model of necroptosis-associated survival using 7 lncRNAs (AC004812.2, AC022915.1, AC073073.2, AC090559.1, AL512330.1, DDN-AS1, and SENCR) in OS. These 7 NRlncRNAs may serve as novel targets for OS treatment and as a more accurate and individualized prognostic monitoring approach.

## Figures and Tables

**Figure 1:** NRlncRNA selection using Lasso mode. (a) Lasso coefficient values for 13 NRlncRNAs in osteosarcoma. The dashed vertical lines represent the optimal log (lambda) value. (b) Lasso coefficient profiles.

**Figure 2:** Screening of prognostic NRlncRNA in OS. (a) Network of lncRNAs and NRlncRNAs coexpressed in OS. (b) An illustration of the association between NRlncRNA, mRNA, and risk types.

**Figure 3:** The KM survival curve. (a) Based on seven NRlncRNAs, the KM survival curve of risk score. (b‑h) The KM survival curves for osteosarcoma patients in various groups.

**Figure 4:** Evaluation of the predictive survival mode of the 7 NRlncRNAs in OS. (a) The UCRA risk score (RS) and clinical factors. (b) MCRA outcomes for RS and CFs. (c) The AUC for RS and CFs, as well as the ROC plots. CFs include gender, M (metastatic), metastasis site, primary tumor site, and specific tumor site.

**Figure 5:** The nomogram of RS and CFs.

**Figure 6:** (a) One-, three-, and five-year ROC plots. (b) An assessment of the association between the predicted and actual OS for the prognostic model using calibration plots. It indicates excellent calibration because the predictive probabilities match the actual probabilities.

**Figure 7:** The outcomes of functional analyses based on NRlncRNAs. (a) GO enrichment analyses. (b) KEGG enrichment analyses.

**Table 1:** Multivariate Cox outcomes of lncRNAs.

lncRNA	Coefficient	HR	95% CI of HR
DDN-AS1	1.501	4.49	2.43-8.28
AC022915.1	-0.665	0.51	0.25-1.08
AC090559.1	-0.566	0.57	0.36-0.89
AL512330.1	0.435	1.55	0.92-2.58
SENCR	0.383	1.47	1.17-1.84
AC073073.2	-0.856	0.42	0.20-0.90
AC004812.2	-1.030	0.36	0.18-0.71

## Data Availability

The datasets used to support the findings of this study are available from TCGA (https://cancergenome.nih.gov/) database.
